The article "Application of Cross-Linked and Non-Cross-Linked Hyaluronic Acid Nano-Needles in Cosmetic Surgery" was retracted in 2023. Reasons: signs of a paper mill; compromised peer review; unreliable results or conclusions.

# Application of Cross-Linked and Non-Cross-Linked Hyaluronic Acid Nano-Needles in Cosmetic Surgery

**DOI:** 10.1155/2022/4565260

**Published:** 2022-05-23

**Authors:** Yiming Huang, Ping Yang

**Affiliations:** Gansu Provincial Maternity and Child-care Hospital, Lanzhou, Gansu 730050, China

## Abstract

The common feature of non-cross-linked hyaluronic acid nano-needles is that they penetrate the skin and dissolve rapidly, and the non-cross-linked hyaluronic acid will migrate under the skin, so it is difficult to maintain the long-term expansion effect in a fixed position. In order to achieve the relatively long-term antiwrinkle effect, a kind of cross-linked and non-cross-linked compound hyaluronic acid microne was prepared. By inserting the microne under the skin, dissolving the non-cross-linked part under the skin and introducing the cross-linked gel particles under the skin, the effect of extending the microne was achieved. The mechanical properties, permeability, and degradation rate of cross-linked and non-cross-linked hyaluronic acid composite nano-needles were studied in detail. Experimental results show that the higher the content of CHA, the slower the degradation rate of the microneedle, and the skin swelling of the HA_CHA (1 : 1) microneedle is the most lasting. With the increase of CHA content in microneedle matrix materials, the degree of epidermal expansion decreased. The preparation of cross-linked and non-cross-linked hyaluronic acid microneedles has the potential to be effectively used as dermal fillers in cosmetics or antiaging treatments.

## 1. Introduction

Hyaluronic acid (HA) is a kind of macromolecular anionic polymer existing in the biological body, which is widely used in medicine, the cosmetics industry, and other biomedical applications [1]. It is endogenous, biocompatible, hydrophilic, viscoelastic, well tolerated, and therapeutic. It is a good barrier inflammatory process and marks the diagnosis of many diseases. The effects of free radicals can prevent and reduce apoptosis and stimulation on proteoglycan, which is very important in the field of cosmetics materials. It has good moisture resistance and locks in water. HA and its derivative sodium hyaluronate are two of the most common cosmetic ingredients, often found in beauty cream formulations and various facial filler injections, because of their excellent permeability, moisturizing properties, and the ability to increase the relative humidity of the skin [2, 3]. In the current beauty market, the use of soluble beauty microne injections instead of hyaluronic acid is a hot beauty patch, and many brands have produced such products. In spite of this, the cross-linked hyaluronic acid is the common characteristic of a microneedle piercing the subcutaneous and quickly dissolving, and the crosslinking hyaluronic acid will occur in the subcutaneous migration. It is difficult to maintain a fixed position in a long-term expansion effect, therefore, not cross-linked hyaluronic acid microneedles even load a lot of effective composition of beauty for a short period of working time and the effect to maintain for a long time is limited, equivalent to only having the effect of optimization utilization efficiency of active ingredients [4].

The article "Application of Cross-Linked and Non-Cross-Linked Hyaluronic Acid Nano-Needles in Cosmetic Surgery" was retracted in 2023. Reasons: signs of a paper mill; compromised peer review; unreliable results or conclusions.

The mechanical properties, penetration rate, and degradation rate of cross-linked and uncross-linked hyaluronic acid composite microneedles were studied in detail. The specific experiments include the preparation of cross-linked hyaluronic acid and cross-linked gel particles, the measurement of axial force of cross-linked composite microneedles, the cross-linking of hyaluronic acid, the determination of cross-linked composite hyaluronic acid in vitro, and the validation of penetration ability of microneedles in mice. Combined with these experiments, the physical and chemical properties of cross-linked composite microneedle hyaluronic acid were evaluated.

In order to achieve a more effective antiwrinkle effect, the preparation of a kind of crosslinking-the cross-linked composite microneedle hyaluronic acid, the characteristics of the microneedle are in soluble cross-linked hyaluronic acid load in the crosslinking hyaluronic acid particles. By using a microneedle into the subcutaneous, the crosslinking will dissolve in part by subcutaneous cross-linked gel particles into the subcutaneous work, which will prolong the effect of microneedle. Zhao yi, dai xing et al. showed through clinical trials that the introduction of compound solution containing sodium hyaluronate by microacupuncture was safe and effective in the application of facial rejuvenation, and the patients were satisfied with it. By He Huinan, xiao-zhong zhao injection cosmetic material classification, different materials are reviewed in this paper. The history and development trend of cosmetics listed the main injection concept of clinical application and development of cosmetic materials which summarizes the characteristics and differences of different brands of injection material. Putting forward the material also needed to be combined with the choice of appropriate injection technology and reference for the demand of comprehensive principles. Facial rejuvenation in injection cosmetology is the most important component of minimally invasive cosmetic surgery. The development and application injection cosmetology technology largely depends on the development of injection materials. According to Yu jiacui, HA contains hydroxyl, carboxyl, and acetylamino polysaccharide chains. Using various modified crosslinking agents such as PEG2000, PDE, BDDE, and ADH as crosslinking agents, three kinds of cross-linked sodium hyaluronate gel with functional properties can be obtained. It lays a necessary scientific and technical foundation for the research and development of new cross-linked sodium hyaluronate gels, thin films, particles or powder formulations with good biological stability, and excellent physical and chemical properties, which can be used for antiadhesion, soft tissue filling, and slow-release drug carriers.

The article "Application of Cross-Linked and Non-Cross-Linked Hyaluronic Acid Nano-Needles in Cosmetic Surgery" was retracted in 2023. Reasons: signs of a paper mill; compromised peer review; unreliable results or conclusions.

## 2. Research Methods

### 2.1. Experimental Drugs and Instruments

The drugs and instruments required for the experiment are shown in Tables 1 and 2.

### 2.2. Preparation of Cross-Linked and Non-Cross-Linked Composite Hyaluronic Acid Microneedles

Join in CHA reagent solution with about 1.0 g HA powder, and mix thoroughly under 40°C 2 H. After crosslinking, the mixed solution contained unreacted fragments of NaOH, BDDE, and HA. HA can be purified with 95% ethanol. The prepared hydrogel was ground, extruded, and screened with a 300 mesh sieve (gB/t6003.1-2012) to obtain particles with a diameter of less than 50PM.  Figure 1 shows the chemical reaction between CHA reagent and BDDE crosslinker under alkaline conditions. In the reaction process, the open BDDE ring reacts with the −oh group of HA to produce the crosslinking network (hydrogel) [5, 6].

Different research ratios affect the performance of micro HA_CHA microneedle. To explore the optimal proportion of micro HA_CHA microneedle two different formulas were adopted, HA and CHA (HA_CHA) ratio (1 : 1) and (5), respectively. Two different weight ratios of formulas are used in the preparation of the HA_CHA microneedle, which (1-0) and the ratio of (1-0) indicating respectively with HA and CHA as a single substrate material of the microneedle. The mixture of polymers with different weight ratios was dissolved in ultrapure water and stirred at 360 RPM with a magnetic stirrer at the room temperature to obtain a homogeneous viscous polymer solution with a concentration of 20% (W/V), in which the suspension containing CHA particles were homogeneous; that is, the particles were evenly distributed in the solution.

### 2.3. Determination of Axial Strength and In Vitro Penetration Ability

The microneedle is compressed vertically between two parallel metal plates of the dynamometer. The single microneedle (height 650PM) was placed on a horizontal platform, and then the stress was applied vertically by a dynamometer probe at a speed of 0.5_/Min. When the probe touched the peak of the microneedle, the testing machine began to show the compression force, and the data was analyzed using the mask-10 software.

The article "Application of Cross-Linked and Non-Cross-Linked Hyaluronic Acid Nano-Needles in Cosmetic Surgery" was retracted in 2023. Reasons: signs of a paper mill; compromised peer review; unreliable results or conclusions.

Insert the microneedle patch into the pig's isolated skin. Use a disposable razor to carefully remove skin hair. Pig isolated skin was purchased from a local slaughterhouse (Beijing, China) and separated into lOcmXlOcm squares with a medical scalpel. Pig isolated skin without subcutaneous tissue samples can be used as a human skin model similarly. HA and 5X5HA_CHA microneedle patches containing different proportions of CHA particles were inserted into the pig's skin in vitro for 5 s and then removed. Then, sulfonyl rhodamine B (model drug) solution was applied to the microneedle insertion site on the skin for 2 Min. Next, the drug sulfonyl rhodamine B, which is not attached to the pinhole on the skin surface, is sucked out. After drying the unabsorbed drug solution on the surface, the array of pinholes containing fluorescence in the skin sample was observed under a fluorescence microscope to evaluate the insertion ability of the microneedle.

### 2.4. In Vivo Effect Verification of Microneedle Mice

The experimental animals were female BALB/C mice with a weight of 20 ± 2 g. It takes about two weeks to acclimatize an animal to laboratory conditions before any experiment to ensure that the experimental conditions remain the same for each mouse. All experiments are approved by the animal health and animal research committee of Beijing University of Chemical Technology and are conducted in accordance with the guiding principles of the experimental animal center of Beijing University of Chemical Technology [7–9]. The experimental process of the animal experiment was as follows: mice were anesthetized with an inhalation anesthesia machine for small animals, and mice were anesthetized with 2.5% isoflurane. Next, use the electric shaver to remove the hair on the back of the mouse on the experimental site needed for the experiment, and use the depilating cream to keep the skin on the back clean. The prepared HA_CHA microneedles were manually inserted into different parts of the mouse back skin, and the microneedles were completely dissolved under the skin after 5 minutes. The handheld digital microscope was used to observe the degree and duration of skin expansion and to evaluate the retention time of microacupuncture effect.

The epidermis of mice after microneedle injection was frozen. The crosslinked hyaluronic acid microneedles of sulfonyl rhodamine B were implanted into the back of mice for smooth hair removal. After 5 minutes, the base was removed, the skin and subcutaneous fat layer of the mice were taken out with a scalpel and quickly frozen with liquid nitrogen. Then, the scalpel is used to slice longitudinally, observe and measure the depth of the subcutaneous puncture needle hole of the mouse with a microscope, and record the puncture depth.

The article "Application of Cross-Linked and Non-Cross-Linked Hyaluronic Acid Nano-Needles in Cosmetic Surgery" was retracted in 2023. Reasons: signs of a paper mill; compromised peer review; unreliable results or conclusions.

## 3. Experimental Results and Analysis

### 3.1. Measurement of Microneedle Axial Strength and In Vitro Microacupuncture Penetration Ability

Figure 2 shows the mechanical behavior (force-displacement curve) of microneedles based on different matrix materials [5, 10, 11]. The data in the figure clearly show that the forces-displacement curve of the microneedle based on the simple non-cross-linked HA (1 : 0) has the highest bending strength, and all of the microneedles with these ratios have excellent mechanical strength. However, due to the different proportions, the internal homogeneous structure of different types of microneedles is different, and the force-displacement curve decreases with the decrease of HA content or the increment of CHA particles in the polymer matrix of microneedles. The different structures of HA and CHA in the HA_CHA microneedle weaken the mechanical stability of the microneedle [8, 12]. The study also showed that the mechanical properties of the microneedle with a heterogeneous structure decreased with the increase of the proportion of mixed particles; however, only a small amount of mechanical properties were enough to penetrate the skin. Therefore, although the mechanical performance of HA_CHA (1 : 1) is lower than that of other mechanical strengths, it still has a certain mechanical strength. Therefore, the prepared HA and ha_cha-based microneedles with different proportions have sufficient insertion capacity in the skin [13–15].

Skin penetration was determined using prepared HA and different proportions of ha_cha-based microneedles, and sulfonyl rhodamine B was used as a model drug for demonstrating skin penetration. Figure 2 shows the luminescence and fluorescence microscopic images after inserting microneedles with different proportions. The fluorescence intensity of HA_CHA (5:1) and HA_CHA (1:0) is roughly the same, which can basically penetrate the skin and has strong mechanical properties. The fluorescence intensity of HA_CHA (1:1) microneedles is slightly weak, which may be because the insoluble particles released into the skin affect the fluorescence absorption of sulfonylrhodamine B by the pinhole, but obvious pores can still be observed, indicating that HA_CHA (1:1) microneedles can completely penetrate the skin. These data show that the proportion of microneedles has little effect on the mechanical properties of microneedles, and the three types of microneedles have sufficient insertion ability.

The article "Application of Cross-Linked and Non-Cross-Linked Hyaluronic Acid Nano-Needles in Cosmetic Surgery" was retracted in 2023. Reasons: signs of a paper mill; compromised peer review; unreliable results or conclusions.

### 3.2. Microneedle Effect in Mice

The in vivo expansion of mouse skin with different HA_CHA ratio was different. All the microneedles with different ratios had sufficient insertion capacity to puncture the mouse epidermis, which was also consistent with the results obtained from the experiments on mechanical strength and skin permeability in vitro. In the first hour after the puncture experiment, HA in the microneedle played an expansion role, and the epidermal expansion reached the maximum. During the first hour of the experiment, the relative epidermal expansion sizes of different polymer-based microneedle arrays were as follows: HA microneedle > HA_CHA (5 : L) microneedle > HA_CHA (1 : 1) microneedle. However, using microneedle skin expansion based on HA gradually disappears in the two days of the experiment, which shows that the HA molecules are fully biodegradable, thus the skin expansion disappears. This is the first in three kinds of microneedle inflation disappearance. It also showed that the pure HA as a substrate material based microneedle's lasting effect is the weakest. In the microneedle based on HA_CHA (5 : 1), the expansion time remained moderate, and basically disappeared on the fourth day of the experiment. However, in the observation of epidermal expansion of mice treated with HA_CHA (1 : 1) microneedle, the epidermal expansion was stable for 4 days and was completely eliminated in the 6-days of the experiment, proving that the skin expansion of HA_CHA (1 : 1) microneedle remained the most persistent. With the increase of CHA content in microneedle matrix materials, the degree of epidermal expansion decreased. By the above experimental phenomena it can be concluded that the expansion of the microneedle into subcutaneous situation depends mainly on CHA crosslinking and reducing water adsorption capacity, and the network structure of CHA limits the expansion of microneedle under the skin; that is, the higher the content of CHA, the lower the content of HA, the expansion of the volume is smaller, but longer the time is needed to maintain the inflation. Compared with the results of the above experiments, the data obtained in vivo were consistent with those obtained in vitro. The expansion of HA_CHA microneedles with different proportions varied, while the higher stability or lower degradation rate of HA_CHA (1 : 1) microneedles showed the potential of matrix materials for skin fillers or antiaging applications.

The microneedle penetrated the skin of the mice, and the insertion depth of the microneedle with a height of 60 (HiM HA) was about 350 | iM under the skin of the mice, and the epidermal layer of the mice had been penetrated by the microneedle. The penetration of the microneedle is effective and allows the microneedle to act under the skin. Therefore, the expansion effect of mouse epidermis was caused by the penetration and dissolution of the microne under the premise that the microne had been penetrated to sufficient depth [16–18].

The article "Application of Cross-Linked and Non-Cross-Linked Hyaluronic Acid Nano-Needles in Cosmetic Surgery" was retracted in 2023. Reasons: signs of a paper mill; compromised peer review; unreliable results or conclusions.

## 4. Conclusion

In this study, the preparation and physicochemical properties of cross-linked and uncross-linked hyaluronic acid composite microne were experimentally verified, and the cross-linked and uncross-linked hyaluronic acid composite microne was explored. Different influencing conditions and controlling factors were used to measure the axial force of cross-linked and non-cross-linked hyaluronic acid microne and the penetration ability of cross-linked and non-cross-linked hyaluronic acid microne in vitro, as well as to verify the effect of microne in vivo. The conclusion of the experiment is that for the proportion of HA_CHA microneedles, the formula has little effect on the mechanical properties of the microneedles, and the three microneedles have sufficient insertion ability on the pig skin in vitro; that is, the three microneedles have excellent mechanical properties. In vitro enzymatic hydrolysis experiments showed that the higher the content of CHA, the slower the degradation rate of microneedle. HA_CHA (1 : 1) microneedles maintained the most persistent skin swelling. With the increase of CHA content in microneedle matrix materials, the degree of epidermal expansion decreased. By the above experimental phenomena it can be concluded that the expansion of the microneedle into subcutaneous situations depends mainly on CHA crosslinking and reduced water adsorption capacity, and the network structure of CHA limits the expansion of microneedle under the skin; that is, the higher the content of CHA, the lower the content of HA. The expansion of the volume is smaller, but a longer time to maintain the inflation is needed. From the above experimental results, it can be seen that the preparation of cross-linked and non-cross-linked compound hyaluronic acid microacupuncture has the potential to be used as an effective dermal filler in cosmetics or antiaging therapy.

## Figures and Tables

**Figure 1:** Chemical reaction equation for the preparation of CHA by BODE crosslinking agent.

**Figure 2:** Axial mechanical strength of HA_CHA microneedles with different proportions.

**Table 1:** Names and specifications of used pharmaceutical reagents.

Drug name	Specifications
Sulfonyl rhodamine B	75%
Sodium hyaluronate	MW = 447.37 nDA
Polydimethylsiloxane	99.5%
Phosphate buffer	Sterile
Ehrlich	>99%
Heavy water	>99.9%
Sucrose	>99.0%
Vitamin C	95%
Coenzyme Q10	95%
Vitamin A palmitate	95%
Poly (PVC)	>79%
Polylactic acid	50–60 kDA
Ethanol	95%
Acetone	99.5%
Isoflurane	100 ML/bottle
1,4-Butanediol glycidyl glycol	MW = 202.25 DA
Oil ether	
Potassium hydroxide	2 MoL/L Aqueous solution
Glacial acetic acid	99.5%
Sodium carbonate	>99.0%
Hyaluronidase	≧300 units/Mg
Physiological saline	For mammals only
Trypan blue	60%
Citric acid-sodium citrate is slow	1 MoL/L, PH = 4.2−
Polylactic acid	50–60 kDA

The article "Application of Cross-Linked and Non-Cross-Linked Hyaluronic Acid Nano-Needles in Cosmetic Surgery" was retracted in 2023. Reasons: signs of a paper mill; compromised peer review; unreliable results or conclusions.

**Table 2:** Names and models of instruments used.

The name of the instrument	Model
Ultrasonic cleaner	BXXW-30AL
Laser etching machine	VLs3.5, 50 W
Digital viscometer	nDJ-9s
The centrifuge	5702RH
Vacuum drying oven	DZF-6050
Vertical flow clean bench	sW-CJ-ZF
Enzyme standard instrument	FL
Handheld digital microscope	AD7013MZt
	□CoRPoRAtion
Fluorescence microscope	sZX7
Ultrapure water machine	XYE-5-H
Dynamometer	MARk-10
Inhalation anesthesia machine	VMR
Vacuum freeze dryer	VFD-1000
Glucose monitor	Easy type

## Data Availability

The data used to support the findings of this study are available from the corresponding author upon request.
